# Polysaccharides from *Rhizoma Atractylodis Macrocephalae*: A Review on Their Extraction, Purification, Structure, and Bioactivities

**DOI:** 10.1155/2022/2338533

**Published:** 2022-08-17

**Authors:** Lei Luo, Jin Cai, Zhang Zhou, Wenqian Tang, Juan Xue, Jinxin Liu, Hongfei Hu, Fan Yang

**Affiliations:** ^1^Department of Health Management Center, Hubei Provincial Hospital of Traditional Chinese Medicine, Wuhan 430070, China; ^2^Department of Hepatobiliary Surgery, The Second People's Hospital of China Three Gorges University, Yichang 443000, China; ^3^Department of Anesthesiology, Wuhan Fourth Hospital, Puai Hospital, Tongji Medical College, Huazhong University of Science and Technology, Wuhan 430035, China; ^4^Department of Gastroenterology, Hubei Provincial Hospital of Traditional Chinese and Western Medicine, Wuhan 430015, China; ^5^School of Clinical Medical, Hubei University of Chinese Medicine, Wuhan 443000, China

## Abstract

*Rhizoma Atractylodes macrocephala* polysaccharide (RAMP), the main bioactive compound extracted from *Rhizoma Atractylodes macrocephala* (RAM), exhibits various biological activities in *in vivo* and *in vitro* methods, such as anti-inflammatory, antioxidant, antitumor, immunomodulatory, hepatoprotective effects, and other functions. This review systematically summarizes the recent research progress on the extraction, purification, structural characteristics, and biological activities of RAMP. We hope to provide a theoretical basis for further research on the application of RAMP in the fields of biomedicine and food.

## 1. Introduction

*Atractylodis macrocephalae* Koidz., known in Chinese as “Bai Zhu,” is a perennial herb belonging to the genus *Compositae* and widely distributed in China, Japan, and Korea [1]. As an important traditional Chinese medicine (TCM), the Rhizome from *Atractylodis macrocephalae* Koidz. (RAM; Figure 1) has been widely used for many years and is mainly distributed in mountainous wetlands, such as Sichuan, Yunnan, and Guizhou in China. TCM holds that RAM is bitter, sweet, and warm and treats a variety of diseases, including abdominal distension, loss of appetite, dizziness, upset, fetal movement, and spontaneous sweating [2–4]. Additionally, the functions of strengthening the spleen and Qi, eliminating dampness, calming the fetus, and promoting diuresis of RAM were recorded by Chinese pharmacopeia (2010) [5]. With an increasing number of modern chemical and pharmacological studies on RAM, it has been found that RAM has anti-inflammatory, antitumor, antioxidant, immune-regulating, antiaging, intestinal function improvement, neuroprotection, and antiuterine contraction effects [6–9]. These pharmacological effects are attributed to its various biologically active ingredients, including steroids, benzoquinones, polysaccharides, coumarins, phenylpropanoids, polyacetylenes, triterpenes, sesquiterpenes, and other chemical substances [10, 11].

Polysaccharides are polymeric carbohydrate composed of at least 10 monosaccharides linked by glycosidic bonds [12]. As we all know, plant polysaccharides, such as pumpkin polysaccharides [13], *Panax ginseng* C. A. Meyer Polysaccharides [14], *Dioscorea* spp. Polysaccharides [15], and Angelica sinensis (Oliv.) Diels polysaccharides [16], have become a new research hotspot in recent years because of their high biological activity and low toxicity. Similarly, as the main active component of RAM, RAM polysaccharide (RAMP) has also attracted increasing attention because of its abundance and diverse bioactivities. Different extraction and purification methods are used to obtain RAMP with different structures and biological activities, and they have been found to have various pharmacological effects, such as antitumor, anti-inflammatory, liver protection, gastrointestinal mucosal protection, and antioxidant effects [17–19].

There is no systematic report on RAMP in the existing literature. In this article, we collected and summarized the contents of RAMP from previous reports and reviewed its extraction method, purification, structure, and biological activity to provide a theoretical basis for further research on the role of RAMP in biomedicine and food fields.

## 2. Extraction and Purification Methods of RAMP

RAMP is a kind of high-molecular-weight compound, and the best method should be selected to facilitate its extraction and purification. However, different extraction temperatures, extraction times, extraction times, and ratios of raw materials to solution and pH values will affect the yield of RAMP. In the past few decades, with the development of technology, the extraction and purification methods of RAMP have been continuously optimized. The flowchart of the extraction, purification, and analysis of RAMP is shown in Figure 2.

### 2.1. Extraction

Conventionally, the water extraction method at a certain temperature has been the most common and classic method used to extract RAMP in the past few decades [20–22]. To more effectively separate RAMP without destroying its structure, different solvent extraction methods and ethanol precipitation methods are often used. Li et al. [23] used hot water extraction and ethanol precipitation methods to separate crude polysaccharide RAMP from the dried rhizome of *Atractylodis macrocephalae* with a yield of 9.65% (w/w). Another experiment mixed 200 g of RAM powder with 2 L of cold water at 4°C to extract RAMP [24]. This method has strong operability, economy, and environmental protection. However, different water extraction conditions, such as extraction time, extraction temperature, source of RAM, and extraction times, may affect the extraction rate and purity of RAMP. In addition, the water extraction method has disadvantages, such as high temperature, long extraction time, low efficiency, and possible degradation of polysaccharides [25].

To improve the extraction efficiency of polysaccharides, other extraction techniques have also been used to extract polysaccharides, such as ultrasonic-assisted extraction and enzyme-assisted extraction. Ultrasonic-assisted extraction has the advantages of energy savings and rapidity and has little effect on the biological activity of polysaccharides [26]. Enzyme-assisted extraction uses special enzymes such as protease and cellulase to destroy the cell wall to promote the release of cell contents, and this method is an efficient and environmentally friendly method [27]. Pu et al. designed an extraction method aimed at further improving RAMP by combining the advantages of ultrasonic-assisted extraction and enzyme-assisted extraction, namely, ultrasonic-assisted enzymatic method [28]. Under the conditions of an extraction temperature of 59.92°C, extraction time of 90.54 min, cellulase concentration of 1.95%, and ultrasonic power of 225.29 W, the yield of crude polysaccharide RAMP was 13.73%. This method has the advantages of time savings and high efficiency.

### 2.2. Purification

Generally, crude polysaccharides obtained through a simple extraction process contain impurities, such as pigments and proteins. If these impurities are not completely removed, they may affect the analysis of polysaccharide structures and the establishment of structure-function correlations. Therefore, further separation and purification of crude polysaccharides to obtain high-quality polysaccharides is an essential step in the analysis and research of polysaccharides. The main purification includes decolorization, deproteinization, and component separation. The common purification methods of polysaccharides include ultrafiltration, ion exchange chromatography, precipitation, macroporous resin column chromatography, and so on.

The Sevag method is a common method for removing protein from crude polysaccharides [29, 30]. In addition, the trichloroacetic acid method and column chromatography method can also be used to remove protein, pigment, and other impurities in crude polysaccharides. For example, Liu et al. [31] used the trichloroacetic acid method to remove the protein, further purified it by DEAE cellulose-52 (2.5 cm × 30 cm) column chromatography and eluted it with distilled water (5 ml/tube). The eluate containing polysaccharide was mixed, concentrated, and lyophilized to obtain purified *Atractylodes macrocephala* polysaccharide (AMP), and the carbohydrate content was 84% as determined by the phenol-sulfuric acid method. The crude polysaccharides were pretreated with papain and further deproteinized by the Sevag method, and the obtained three polysaccharides, RAMP70, RAMP80, and RAMPtp, were detected with carbohydrate contents of 96.05%, 97.67%, and 95.66%, respectively [32]. In addition, the ultrafiltration membrane method was also used to purify RAMP [33]. Use 150 ml of ethanol to precipitate the crude polysaccharide supernatant by Sevag method to remove protein, store at 4°C for 2 h, take the supernatant, add 750 mL of ethanol to precipitate, and store at 4°C for 2 h. The obtained precipitate was dissolved in 20 ml of ultrapure water and centrifuged at 12000 rpm for 10 min. The supernatant was collected and dialyzed for two days and purified by 5KD ultrafiltration membrane to obtain RAMP [24]. The results showed that the total polysaccharide content in RAMP was 96.47%. Cui et al. [34] purified three water-soluble polysaccharides from RAM by a combination of ion exchange and gel permeation column chromatography. The yields of AMAP-1, AMAP-2, and AMAP-3 were 11.8% (353.8 mg), 6.8% (203.9 mg), and 5.6% (166.5 mg), respectively.

## 3. Physiochemical and Structural Features of RAMP

Polysaccharide has a variety of pharmacological effects, and its structural characteristics (including molecular weight, the type, position and configuration of glycosidic bond, and composition of monosaccharide) are the key to determining its pharmacological effects, so it is of great significance to study its structural characteristics. The basic structure, molecular weight, and monosaccharide composition of RAMP were reported mainly by high performance gel permeation chromatography (HPGPC), gas chromatography-mass spectrometry (GC-MS), nuclear magnetic resonance (NMR), high performance liquid chromatography (HPLC), periodic acid oxidation, Smith degradation, and infrared spectroscopy.  Table 1 summarizes the molecular weight and possible structure of RAMP.

### 3.1. Average Molecular Weights

HPGPC and HPLC are the main methods for determining the average molecular weight of RAMP [35, 36]. Xue et al. [37] extracted two polysaccharides RAMP1 and RAMP2 from *Atractylodes Rhizoma* and measured their molecular weights to be 1.851 × 10^6^ Da and 4.354 × 103 Da, respectively. Another study [38] used a GPC-RI-MALS instrument (gel chromatography-differential-multiangle laser light scattering) to determine the average molecular weight of RAMP to be 4.748 × 103 Da. However, due to the different origins and extraction methods of *Atractylodis macrocephalae*, the average molecular weight of RAMP is different. Wang et al. [39] measured the molecular weight of RAMP by HPGPC methods to be 28773 Da.

### 3.2. Monosaccharide Compositions

In general, after the polysaccharide is completely acid hydrolyzed by strong acid reagents such as hydrochloric acid and trifluoroacetic acid at a certain temperature, the composition of the monosaccharide can be obtained by ion chromatography (IC), gas chromatography (GC), and HPLC. The component analysis of monosaccharides can be used to further analyse the structure of polysaccharides and plays an important role in the research or production of polysaccharide drugs [40].

Polysaccharides composed of two or more different monosaccharide molecules are called heteropolysaccharides [41]. Feng et al. [24] obtained a polysaccharide RAMP from RAM by cold water extraction, ethanol precipitation, and ultrafiltration membrane purification. Then, the monosaccharide composition of RAMP was determined by trifluoroacetic acid hydrolysis and gas chromatography, and it was found that RAMP was a neutral heteropolysaccharide composed of arabinose (Ara), glucose (Glc), and galactose (Gal) in the ratio of 1.5 : 5:1. Another study [38] used IC methods to determine that RAMP is mainly composed of Glc, Gal, Ara, fructose (Fru) and mannose (Man), accounting for 67.01%, 12.32%, 9.89%, 1.18%, and 0.91%, respectively. It has been reported that glucose is the main component of most RAMP, but the composition and proportion of other components are different. The composition of monosaccharides is shown in Table 1.

### 3.3. Chemical Structures

Except for the molecular weight and monosaccharide composition, the structural features of RAMP were elucidated by methylation, periodate oxidation, Smith degradation, NMR, and ^13^C and ^1^H. Some previous studies have reported the possible structure of RAMP and the backbones and branches of which are summarized in detail in Table 1. Studies [42] have confirmed that RAMP is a polysaccharide with *α* and *β* configurations by infrared spectroscopy (FTIR) and hydrogen nuclear magnetic resonance spectroscopy (^1^H NMR), but the *β* configuration is dominant. Lin et al. [43] extracted an inulin-type polysaccharide from *Atractylodes Rhizoma* and then used electrospray ionization mass spectrometry (ESI-MS), NMR, and hydrophilic interaction liquid chromatography (HILIC) method to study its structure and found that the main chain of RAMP is composed of a-D-Glcp-[-(1 ⟶ 2)-*β*-D-Fruf-]_8_-(1 ⟶ 2)-*β*-D-Fruf. The NMR results suggested that RAMP2 contained a backbone chain mainly consisting of ⟶ 3-*β*-D-Glcp-(1 ⟶, ⟶ 3, 6-*β*-D-Glcp-(1 ⟶, ⟶ 6-*β*-D-Glcp-(1 ⟶, T-*β*-D-Glcp, ⟶ 4-*α*- GalpA-(1 ⟶, ⟶ 4-*α*-GalpA-OMe-(1 ⟶, ⟶ 5-*α*-Araf-(1 ⟶, ⟶ 4, 6-*β*-manp-(1 ⟶  and ⟶ 4-*β*-Galp-(1 ⟶  [37].

### 3.4. Molecular Morphology

The molecular morphology of polysaccharides is closely related to the understanding of their pharmacological activities. To fully understand the molecular morphology of RAMP, scanning electron microscopy (SEM), atomic force microscopy (AFM), and transmission electron microscopy (TEM) were used to study the microstructure of these macromolecules (Figure 3). Through the observation of RAMP, it was found that the diameter of RAMP molecule is 42.2 nm, the morphology of molecular chain is an inding coil and spherical distribution, and multiple nodular polysaccharides are combined with each other through intermolecular interactions [39]. Another study also confirmed that RAMP is a spherical structure with a clastic petal like texture on the surface [37]. Under the condition of high vacuum, the images of RAMPtp were obtained by SEM with different multiples (1000, 2000, 5000, 10000, 20000, and 30000 times) and found that RAMPtp was oval-shaped particles with relatively smooth surface and complex polymer network structure [32].

## 4. Biological Activities

### 4.1. Gastrointestinal Tract Protection Activities

In recent years, plant polysaccharides, such as ginseng polysaccharides and poria cocos polysaccharide, have received extensive attention due to their role in regulating gut microbes [44, 45]. In traditional Chinese medicine, RAM is used to treat abdominal distension, diarrhea, and anorexia because it has the function of strengthening the spleen and stopping diarrhea. As one of its active ingredients, the study of ERIC-PACR fingerprints showed that RAMP could improve the flora of intestinal disorders and could be used as an oral adjuvant for the regulation of intestinal flora [39]. In a study of LPS-induced gosling enteritis, it was found that RAMP increased the levels of intestinal tight junction proteins occludin and ZO-1 and improved intestinal flora disturbance, thereby relieving gosling enteritis [46]. Gut microbiota metabolites, such as short-chain fatty acids and secondary bile acids, are important factors in the development of a variety of intestinal diseases [47]. In the experiment of dextran sulfate sodium- (DSS-) induced ulcerative colitis (UC) in mice, it was shown that RAMP could improve the damage of colon and regulate the metabolic levels of short-chain fatty acids and bile acids, which provided a new possibility for the clinical treatment of UC [48]. Dan et al. found that RAMP could significantly increase the polyamine content, cytoplasmic Ca2^+^ level, promote cell migration, and increase Kv1.1 mRNA and protein expression in IEC-6 cells. These effects suggested that RAMP significantly promotes the migration of intestinal epithelial cells by activating the polyamine-kv1.1 signaling pathway, which may promote the healing of intestinal injury [49].

### 4.2. Hepatoprotective Activities

It has been reported that many factors, such as hyperlipidemia, alcohol consumption, drug abuse, and hepatitis virus infection, can lead to liver injury [50, 51]. Several studies have shown that RAMP has a hepatoprotective effect and the mechanism is mainly attributed to its antioxidant, anti-inflammatory, and lipid metabolism regulation [21, 22]. Guo et al. [38] reported that RAMP has a protective effect on LPS-induced acute liver injury and mainly by activating the TLR4-MyD88 signaling pathway, reducing the levels of interleukin-1*β* (IL-1*β*), interleukin-6 (IL-6) and tumor necrosis factor-*α* (TNF-*α*), and inhibiting the expression of glutathione peroxidase (GSH-PX) and malondialdehyde (MDA). This indicated that the liver protective effect of RAMP is mainly achieved by reducing inflammatory damage and oxidative stress. Another study [52] also found that RAMP, a homogeneous polysaccharide isolated and purified from *Atractylodes Rhizoma*, had a hepatoprotective effect on carbon tetrachloride- (CCl4-) induced mouse liver injury model. RAMP could reduce the activity of nitric oxide synthase (NOS) and the content of nitric oxide (NO) and MDA in liver tissue and increase the activities of superoxide dismutase (SOD) and GSH-PX, showing that RAMP achieves liver protection through antioxidant effects. In addition, RAMP was used to reduce hepatic TG content and regulate hepatic lipid metabolism, which provided the possibility for the clinical treatment of nonalcoholic fatty liver disease [53].

### 4.3. Antitumor Activities

*In vivo* and *in vitro* experiments confirmed that RAMP has potential antitumor activity. *In vitro* experiment [33] found that RAMP at a dose of 2 mg/mL inhibited the proliferation of human esophageal cancer Eca109 cells by 74.63%. Furthermore, annexin V/PI staining showed that the fluorescence intensity of Eca109 cells decreased with the increasing of RAMP concentration. Meanwhile, western blot analysis showed that RAMP could lead to a decrease in the expression of the anti-apoptotic protein Bcl-2 and an increase in the expression of Bax, cytochrome C, and caspases 9 and 3 in Eca-109 cells. These results showed that RAMP could inhibit the growth of Eca109 cells and induce Eca109 cell apoptosis. In a study of the antitumor effect of RAMP on glioma C6 cells, Li et al. [23] also confirmed that RAMP could induce C6 cell death by inducing apoptosis and induce cell death by activating caspases 9 and 3 and PARP cleavage apoptosis. By seeding H22 tumor cells into mice, treatment with RAMP was found to inhibit tumor growth while promoting T cell expression, thereby exerting an antitumor effect [24]. In addition, Feng et al. [54] demonstrated for the first time that RAMP could activate macrophages through the TLR4/MyD88 pathway to exert the effect of antitumor activity, which provided the possibility for RAMP to become a potential drug for tumor immunotherapy.

### 4.4. Immunomodulatory Activities

Immune regulation is the key for the body to maintain its own physiological stability. In recent years, plant polysaccharides have been widely studied for the immunomodulatory effects by regulating cytokines, lymphocytes, antibody levels, and neuroendocrine system [55, 56]. This compound has a low toxicity and is an effective biological response regulator. Similarly, RAMP also showed good immunomodulatory activity in previous studies.

Macrophages play a role in immune defense by phagocytes or secreting cytokines such as NO, TNF-*α*, and interleukin-1 (IL-1) to kill pathogens [57]. RAMP increases the release of NO, ROS, IL-6, interleukin-1 (IL-10), TNF-*α*, and chemokines, enhances pinocytosis and phagocytosis, and induces the activation of macrophages to play an immunoregulatory function [58]. Ji et al. [59] found that RAMP increased the phagocytosis of macrophages in a concentration-dependent manner, and the phagocytosis of macrophages was the strongest at concentrations of 100 *μ*g/ml and 200 *μ*g/ml. In addition, *in vitro* experiments [60] found that RAMP enhanced NK cytotoxicity, promoted splenocyte proliferation, and increased the secretion of NO, IgG, and cytokines. Further study found that RAMP may induce splenocyte activation through TLR4-independent MAPK and NF-*κ*B signaling pathways. An experiment on immunosuppressive geese induced by cyclophosphamide showed that RAMP could reduce the degree of spleen injury, reduce the proliferation of T cells and B cells, reverse the dysfunction of cellular and humoral immunity, and ultimately reduce the immunosuppressive effect [61]. To explore the molecular mechanism of RAMP regulating immune function, through *in vitro* and *in vivo* experiments, Li et al. [62] found that RAMP activates thymic T lymphocytes through the mir2/CTLA4/CD28/AP-1 signaling pathway, promotes the activation and proliferation of T lymphocytes, and maintains the normal morphology of thymocytes to regulate immune function.

### 4.5. Antioxidant and Antiaging Activities

Oxidative stress has been confirmed to be related to the occurrence and development of various diseases, including atherosclerosis, cancer, and diabetes [63]. Meanwhile, it plays an important role in the rate of aging [64]. Natural materials are a promising source of antioxidants, and various bioactive components of fungi, plants, and animals, especially polysaccharides, have antioxidant activity [65, 66]. Polysaccharides play an antioxidant role by inhibiting and scavenging free radicals and increasing the activity of antioxidant enzymes [67, 68]. Multiple studies have shown that RAMP has antioxidant and antiaging activities. We found that RAMP could significantly reduce the activities of MDA and MAO in the serum and brain tissue, increase the activities of SOD, GSH-Px, and catalase (CAT) in serum, and increase the content of total antioxidant capacity (T-AOC) in brain tissue. This indicated that RAMP might play a role in relieving aging by enhancing the body's antioxidant capacity [69]. In addition, we have mentioned earlier that RAMP could reduce oxidative stress in mice by inhibiting the levels of GSH-PX and MDA, thereby protecting the liver [38]. The 1,1-diphenyl-2-pyridyl hydrazide free radical 2,2-diphenyl-1-(2,4,6-trinitrophenyl) (DPPH) scavenging rate was used to represent the antioxidant capacity of RAMP. Pu et al. [28] found that the DPPH scavenging rate of RAMP obtained using the UAEE optimization process was better than that obtained using methods, and the DPPH scavenging rate reached 62.18%. Another study [50] confirmed that RAMP obviously scavenges DPPH, superoxide anions, and hydroxyl free radicals, reduces the activity of NOS and the content of NO and MDA in liver tissue, increases the activities of SOD and glutathione peroxidase (GSH-PX), and shows obvious antioxidant activity *in vitro*.

### 4.6. Other Biological Activities

RAMP also showed neuroprotective activity. To construct the hypoxia model of primary rat cerebral cortical neurons, RAMP significantly inhibited the apoptosis of neurons induced by hypoxia, reduced the damage of mitochondria, downregulated the mRNA and protein expression of apoptotic proteins caspase 3 and Bax, and increased the level of anti-apoptotic protein Bcl-2 [70]. Inflammation is the subsequent response of the body's immune system to injury, infection, and stress. Plant polysaccharides have received increasing attention and research due to their safety and effective anti-inflammatory effects [71]. For example, Liu et al. [72] found that polysaccharides isolated from lignified okra significantly ameliorated LPS-induced inflammatory injury in RAW 264.7 cells by inhibiting NO secretion and reducing the levels of proinflammatory factors (IL-1*β*, iNOS, and TNF-*α*). Meanwhile, an anti-inflammatory effect is an important biological activity of RAMP. Disorder of intestinal function are closely related to the occurrence of inflammation. RAMP could alleviate enteritis by reducing serum levels of IL-1*β*, IL-6, TNF-*α*, and CRP [46]. In addition, study has found that RAMP reduces the inflammatory factor expression of TNF-a and IL-4 in the spleen to improve the immune response [73].

## 5. Conclusion and Future Perspectives

In China, RAM has been used as a traditional Chinese herbal medicine for thousands of years to treat various diseases including spontaneous sweating, loss of appetite, abdominal distension, fetal restlessness, diarrhea, and spleen deficiency. RAMP, as the main active ingredient of RAM, has received more and more research because of its extensive pharmacological effects and biological activities. Previous studies have shown that RAMP is a polar polymer compound with a molecular weight between 2 and 200 KDa that is water-soluble and contains carbohydrates. The water extraction method and the ultrasonic-assisted enzymatic method are the main extraction methods of RAMP. Among them, the ultrasonic-assisted enzymatic method is more effective. However, the yields of RAMP obtained by existing extraction methods are not high. The extracted RAMP usually contains proteins, pigments, and other impurities, which can be purified by ultrafiltration, ion exchange chromatography, precipitation, and macroporous resin column chromatography. Different extraction and purification methods have different RAMP monosaccharide compositions. Therefore, the extraction and purification methods of ASP still need further research.

The structure of polysaccharides is a prerequisite for studying their underlying mechanisms and structure–activity relationships. The structural characteristics of polysaccharides include molecular weight, monosaccharide composition, molecular morphology, glycosidic bond configuration, and so on. Techniques such as HPGPC, FTIR, GC-MS, HPLC, NMR, and FTIR can be used to identify the chemical composition and structure of RAMP. However, recent studies on the structural characteristics of RAMP have mainly focused on molecular weight, monosaccharide composition, and even some primary structures. Only a few RAMPs have identified the types of connecting rods, and their detailed structural features require further study. Meanwhile, due to the different sources of raw materials, extraction methods, and purification techniques, the molecular weight, molecular structure, and spatial conformation of polysaccharides will be changed, and ultimately the biological activities of polysaccharides may be different. Future works should focus on the relationship between the structure and bioactivity of RAMP to enhance our understanding of the functional effects of RAMP.

RAMP has various pharmacological activities, including anti-inflammatory, gastrointestinal protection, antitumor, antioxidant, antiaging, neuroprotective, hepatoprotective, and immunomodulatory effects. The mechanisms of different pharmacological actions are interrelated. Studies have found that the hepatoprotective effect of RAMP involves multiple mechanisms of antioxidant and anti-inflammatory effects. The anti-inflammatory and antiaging properties of RAMP are closely related to immune mechanisms. Therefore, RAMP does not work through a single channel, but multiple mechanisms are interconnected and work together.

RAMP, as the main active ingredient of RAM and involved in multiple biological functions, has huge potential health benefits and broad application prospects in the field of biomedicine. However, research on RAMP has been explored in *in vitro* and *in vivo* experiments, but not in humans. Therefore, further research is needed on the effectiveness and reliability of RAMP in humans. In addition, the application of new research techniques, including metabolomics, microbiomics, proteomics, and bioinformatics, will further help to reveal the biological activity mechanism of RAMP. This paper highly summarizes the extraction, purification, structural characteristics, and pharmacological properties of RAMP and draws the fact that RAMP has become a potential treasure house of drugs and functional foods. With the continuous deepening of human research on RAMP, it is believed that it will have a good prospect and broad market in biomedical and food applications soon.

## Figures and Tables

**Figure 1:** (a) The above-ground part of *Atractylodis macrocephalae* Koidz; (b) medicinal portion of *Atractylodis macrocephalae* Koidz.; (c) commercial herbal pieces of *Rhizoma Atractylodis macrocephalae*.

**Figure 2:** The flowchart of the extraction, purification, and analysis of RAMP.

**Figure 3:** AFM, TEM, and SEM images of *Rhizoma Atractylodis Macrocephalae* polysaccharides [32, 37, 39]. (a) AFM image of of PAM; (b) TEM spectrum of RAMP2 in purified water; (c) the morphology of RAMP2 at 10000×, scale bar = 5 *μ*m; (d) SEM image of RAMPtp at 30000×, scale bar = 1 *μ*m.

**Table 1:** The polysaccharides isolated from *Rhizoma Atractylodes macrocephala*.

NO.	Compound name	Monosaccharide compositions	Molecular weight	Possible structures	Bioactive activities	Reference
1	BZ-3-1	Rha, Ara, Xyl, Man, Glc, and Gal in the ratio of 14.1 : 39.4 : 1.4 : 4.2 : 22.6 : 18.3	5.65 × 10^4^ Da	NA	Immunomodulatory activity	20
2	BZ-3-2	Rha, Ara, Xyl, Man, Glc, and Gal in the ratio of 2.6 : 7.6 : 21.1 : 62.6 : 6.1	5.59 × 10^4^ Da	NA	NA	20
3	BZ-3-3	Man : Glc in the ratio of 15.4 : 85.6	5.51 × 10^4^ Da	NA	NA	20
4	PAMK	Glc and Man in the ratio of 0.582 : 0.418	2.816 KDa	1 ⟶ 6 linked monosaccharide backbone and 1 ⟶ 3 linked signal of glucose residues at the position 3–C	Hepatoprotective	22
5	PAMK	Gal, Ara, and Glc in the ratio of 1 : 1.5 : 5	4.1 KDa	NA	Anti-tumor activity	24
6	RAMPtp	Glc, Man, Rha, Ara, and Gal in the ratio of 60.67 : 12.99 : 10.61 : 8.83 : 4.9	1.867 × 10^3^ KDa	Backbone composed of 1, 3-linked *β*-D Galp and 1, 6-linked *β*-D Galp residues	Immunomodulatory activity	32
7	APA	Ara and Glc in the ratio of 1 : 4.57	2.1 KDa	Composed of pyranose rings and *α*-type and *β*-type glycosidic linkages.	Anti-tumor activity	33
8	AMAP-1	Rha, Ara, Gal, and GalA in the ratio of 10.1 : 18.4 : 26.9 : 44.6	137.5kD	Backbone composed of (1 ⟶ 4)-linked GalpA residues	Immunomodulatory activity	34
9	AMAP-2	Rha, Ara, Gal, and GalA in the ratio of 12.8 : 23.5 : 9.5 : 54.1	161.9kD	Backbone composed of (1 ⟶ 4)-linked GalpA residues	Immunomodulatory activity	34
10	RAMP2	Man, GalA, Glc, Gal, and Ara in the ratio of 1.00 : 8.58 : 27.28 : 3.68 : 4.99	4.354 KDa	Backbone composed of ⟶ 3-*β*-glcp-(1 ⟶ , ⟶ 3,6-*β*-glcp-(1 ⟶ , ⟶ 6-*β*-glcp-(1 ⟶ , T -*β*-glcp-(1 ⟶ , ⟶ 4-*α*-galpA-(1 ⟶ , ⟶ 4-*α*-galpA-6-OMe-(1 ⟶ , ⟶ 5-*α*-araf-(1 ⟶ , ⟶ 4,6-*β*-manp-(1 ⟶ and ⟶ 4-*β*-galp-(1 ⟶	Immunomodulatory activity	37
11	PAMK	Ara, Gal, and Glc in the ratio of 1 : 1.25 : 6.78	4.748 × 10^3^ g/mol	NA	Hepatoprotective and anti-inflammatory activity	38
12	PAM	Rha, Glc, Man, Xyl, and Gal in the ratio of 0.03 : 0.25 : 0.15 : 0.41 : 0.15	28773 Da	NA	Gastrointestinal tract protection activity	39
13	RAMPS	Rib, Ara, Rha, Man, Glu, and Gal in the ratio of 1.0 : 4.3 : 0.1 : 5.7 : 2.8 : 2.2	NA	NA	Gastrointestinal tract protection activity	50
14	PRAM2	Rha, Xyl, Ara, Glc, Man and Gal in the ratio of 1 : 1.3 : 1.5 : 1.8 : 2.1 : 3.2	19.6 KDa	NA	Hepatoprotective, antioxidant, and anti-inflammatory activity	53
15	RAMPS	Glu, Man, Ara, Gal, and Xyl in the ratio of 66.39 : 21.24 : 5.64 : 2.65 : 2.3	109.4 KDa	Backbone composed of 1, 3-linked *β*- D-Galp and 1, 6 –linked *β*-D-Galp residues	Immunomodulatory activity	56
16	AMP	Glc, Gal, Rha, and Man in the ratio of 7.36 : 1.00 : 3.05 : 1.52	8.374 kDa	NA	Immunomodulatory activity	60

NA: information was not available. Glc: glucose; Gal: galactose; Man: mannose; Ara: arabinose; Xyl: xylose; Rha: rhamnose; Glu: glucose; Fru: fructose; Rib: ribose; GalA: galacturonic acid.
